# Prognostic Value of Malondialdehyde Serum Levels in Severe Sepsis: A Multicenter Study

**DOI:** 10.1371/journal.pone.0053741

**Published:** 2013-01-14

**Authors:** Leonardo Lorente, María M. Martín, Pedro Abreu-González, Alberto Domínguez-Rodríguez, Lorenzo Labarta, César Díaz, Jordi Solé-Violán, José Ferreres, Juan María Borreguero-León, Alejandro Jiménez, Armando Morera-Fumero

**Affiliations:** 1 Intensive Care Unit, Hospital Universitario de Canarias, La Laguna, Santa Cruz de Tenerife, Spain; 2 Intensive Care Unit, Hospital Universitario Nuestra Señora de Candelaria, Santa Cruz de Tenerife, Spain; 3 Department of Physiology, Faculty of Medicine, University of the La Laguna, Santa Cruz de Tenerife, Spain; 4 Department of Cardiology, Hospital Universitario de Canarias, Ofra, La Laguna, Santa Cruz de Tenerife, Spain; 5 Intensive Care Unit, Hospital San Jorge de Huesca, Huesca, Spain; 6 Intensive Care Unit, Hospital Insular, Las Palmas de Gran Canaria, Spain; 7 Intensive Care Unit, Hospital Universitario Dr. Negrín, Las Palmas de Gran Canaria, Spain; 8 Intensive Care Unit, Hospital Clínico Universitario de Valencia, Valencia, Spain; 9 Laboratory Department, Hospital Universitario de Canarias, La Laguna, Santa Cruz de Tenerife, Spain; 10 Research Unit, Hospital Universitario de Canarias, La Laguna, Santa Cruz de Tenerife, Spain; 11 Department of Internal Medicine and Psychiatry, Faculty of Medicine, University of the La Laguna, Santa Cruz de Tenerife, Spain; Universidad Peruana Cayetano Heredia, Peru

## Abstract

**Objective:**

The oxidant/antioxidant state in septic patients has only been studied in small series. We wished to determine whether malondialdehyde (MDA) serum levels were associated with severity and 30-day mortality in a large series of patients with sepsis.

**Methods:**

We performed an observational, prospective, multicenter study in six Spanish Intensive Care Units. Serum levels of MDA were measured in a total of 228 patients (145 survivors and 83 non-survivors) with severe sepsis and 100 healthy controls**.**

**Results:**

Serum levels of MDA were higher in severe septic patients than in healthy controls. Non-surviving septic patients had higher MDA values than survivors. MDA serum levels were associated with severity markers (lactic acid, SOFA, APACHE-II) and coagulation indices. Regression analysis showed that MDA serum levels were associated with 30-day survival (Hazard ratio = 1.05; 95% confidence interval = 1.009–1.091; p = 0.016). Receiver operating characteristic analysis showed that the area under curve of MDA serum levels to predict 30-day survival was 0.62 (95% CI = 0.56–0.69; P = 0.002). The risk of death in septic patients with MDA serum levels above 4.11 nmol/mL was higher than in patients with lower values (Hazard Ratio = 2.43; 95% CI = 1.49–3.94; p<0.001).

**Conclusions:**

The novel findings of our study on severe septic patients, to our knowledge the largest series providing data on the oxidative state, are that elevated MDA serum levels probably represent an unbalanced oxidant state and are related with poor prognosis in patients with severe sepsis.

## Introduction

Severe sepsis is a common, resource-consuming and frequently fatal condition, associated with as many deaths annually as acute myocardial infarction [1], [2].

The oxidant and antioxidant state in septic patients has been scarcely assessed and then only in small series [3]–[6]. A higher antioxidant state, determined by different compounds, has been found in non-surviving than in surviving septic patients [4]–[6]. In addition, a study of 12 patients by Ogilvie et al found higher malondialdehyde (MDA) serum levels in non-surviving than in surviving critically ill septic patients [3]; however, the sample size was too small to demonstrate that MDA serum levels could be used as a biomarker to predict clinical outcome of septic patients.

Oxidative damage is a result of an imbalance between oxidants and antioxidants and includes oxidative modification of cellular macromolecules, induction of cell death by apoptosis or necrosis, as well as structural tissue damage. MDA is a low molecular weight aldehyde that results from free radical attacks on polyunsaturated fatty acids. MDA measurement can be considered a valuable screening tool as a biomarker of oxidative damage [7].

Thus, the objective of this study was to determine whether MDA serum levels are associated with severity and early mortality in septic patients and whether these serum levels could be used as biomarkers to predict the clinical outcome of septic patients in a large series of patients.

## Methods

### Design and Subjects

A multicenter, observational, prospective study was carried out in six Spanish Intensive Care Units. The study was approved by the Institutional Review Boards of the six hospitals recruiting patients. All patients provided written informed consent to participate in the study.

Inclusion criteria were the diagnosis of severe sepsis according to the International Sepsis Definitions Conference criteria [8]. Exclusion criteria were: age <18 years, pregnancy, lactation, human immunodeficiency virus (HIV), white blood cell count <1,000/µl, solid or hematological tumor, or immunosuppressive, steroid or radiation therapy. A total of 228 patients with severe sepsis and 100 healthy controls were included.

### Variables Recorded

The following variables were recorded for each patient: sex, age, diabetes mellitus, chronic renal failure (defined as glomerular filtration rate (GFR) <60 ml/mn per 1.73 m^2^), chronic obstructive pulmonary disease (COPD), site of infection, creatinine, leukocytes, lactic acid, platelets, international normalized ratio (INR), activated partial thromboplastin time (aPTT), Acute Physiology and Chronic Health Evaluation II (APACHE II) score [9], Sepsis-related Organ Failure Assessment [SOFA] score [10], tumor necrosis factor (TNF)-alpha, interleukin (IL)-10 and 30-day mortality.

Blood samples were collected from 228 patients with severe sepsis at the time of the diagnosis and from 100 healthy controls.

### MDA Serum Level Analysis

Serum MDA levels were measured using thiobarbituric acid-reactive substance (TBARS) method as described by Kikugawa et al [11]. The pink complex of samples was extracted in n-butanol. Each sample was placed in a 96-well plate and read at 535 nm in a microplate spectrophotometer reader (Benchmark Plus, Bio-Rad, Hercules, CA, USA). The detection limit of this assay was 0.079 nmol/ml; the intra- and inter-assay CV were 1.82% and 4.01%, respectively. The serum concentration of MDA was expressed in nmol/ml. To avoid the possible dispersion of MDA serum level results, all the samples were processed at the same time, at the end of the recruitment process.

### Statistical Methods

In a pilot study with 30 patients with severe sepsis, we found that surviving patients showed lower circulating levels of MDA (3.14±1.22 nmol/mL) than non-survivors (3.65±1.82 nmol/mL). We calculated that 228 patients in a cohort study were needed in order to demonstrate significant differences in the circulating levels of MDA between groups, for a power of 80% and a type I error rate of 5%.

Continuous variables are reported as medians and interquartile ranges. Categorical variables are reported as frequencies and percentages. Comparisons of continuous variables between groups were carried out using Wilcoxon-Mann-Whitney test. Comparisons between groups for categorical variables were carried out with chi-square test. The association between continuous variables was carried out using Spearmańs rank correlation coefficient or Spearman's rho coefficient. We plotted a receiver operating characteristic (ROC) curve using survival at 30 days as classification variable and MDA level as prognostic variable. The cut-off prognostic value of the serum levels of MDA was selected with the likelihood ratio between sensitivity and 1-specificity (likelihood ratio = 2.0). Analysis of survival at 30 days with Kaplan-Meier method curve and comparisons by log-rank test were carried out using MDA serum levels lower/higher than 4.11 nmol/mL as the independent variable and survival at 30 days as the dependent variable. Cox regression analysis was applied to determine the independent contribution of MDA serum levels on the prediction of 30-day mortality. To avoid collinearity effect [12], we only included age, lactic acid, APACHE-II and aPTT as co-predictors. Hazard ratio and 95% confidence intervals were calculated as measures of the clinical impact of the predictor variables. A P value of less than 0.05 was considered statistically significant. Statistical analyses were performed with SPSS 17.0 (SPSS Inc., Chicago, IL, USA) and NCSS 2000 (Kaysville, Utah).

## Results

We found lower MDA serum levels in septic patients than in healthy controls; however, there were no significant differences between both groups in terms of age and sex (Table 1).

**Table 1:** Demographic’ characteristics of healthy controls and septic patients.

	Healthy controls (n = 100)	Septic patients (n = 228)	p-value
Gender male – n (%)	62 (62.0)	150 (65.8)	0.53
Age - median years (p 25–75)	59 (47–70)	60 (48–71)	0.74
MDA - median nmol/mL(p 25–75)	1.11 (0.78–1.51)	3.20 (2.06–4.86)	<0.001

Comparison of demographic and clinical parameters between non-surviving (n = 83) and surviving septic patients (n = 145) are shown in Table 2. No differences were observed regarding sex, chronic renal failure, COPD, diabetes mellitus, ischemic heart disease, site of infection, microorganism responsible, bloodstream infection, antimicrobial treatment and TNF-alpha; however, the non-surviving septic patients showed higher age, higher levels of lactic acid and IL-10 and creatinine, increased SOFA and APACHE-II scores, prolonged aPTT, and reduced platelet count. Moreover, non-surviving patients had higher serum levels of MDA (p = 0.002) than survivors.

**Table 2:** Patients’demographic and clinical characteristics of septic patients.

	Survival (n = 145)	Non-survival (n = 83)	p-value
Gender male – n (%)	94 (64.8)	56 (67.5)	0.77
Age - median years (p 25–75)	55 (44–66)	64 (55–74)	0.001
Diabetes mellitus – n (%)	41 (28.3)	31 (37.3)	0.18
Chronic renal failure – n (%)	8 (5.5)	8 (9.6)	0.28
COPD – n (%)	16 (11.0)	13 (15.7)	0.31
Ischemic heart disease - n (%)	13 (9.0)	6 (7.2)	0.80
Site of infection			0.68
· Respiratory - n (%)	81 (55.9)	48 (57.8)	
· Abdominal - n (%)	39 (26.9)	22 (26.5)	
· Neurological	3 (2.1)	0	
· Urinary - n (%)	8 (5.5)	5 (6.0)	
· Skin - n (%)	8 (5.5)	3 (3.6)	
· Endocarditis - n (%)	6 (4.1)	4 (4.8)	
· Osteomyelitis - n (%)	0	1 (1.2)	
Microorganism responsibles			
· Unkwon - n (%)	77 (53.1)	47 (56.6)	0.68
· Gram-positive- n (%)	32 (22.1)	19 (22.9)	0.87
· Gram-negative- n (%)	35 (24.1)	17 (20.5)	0.62
· Fungii- n (%)	4 (2.8)	4 (4.8)	0.47
· Anaerobe- n (%)	1(0.7)	1 (1.2)	0.99
Bloodstream infection	22 (15.2)	11(13.3)	0.84
Empiric antimicrobial treatment adequate			0.85
· Unkown due to negative cultures- n (%)	77 (53.1)	47 (56.6)	
· Adequate - n (%)	58 (40.0)	31 (37.3)	
· Unkown due to antigenuria diagnosis-n(%)	4 (2.8)	3 (3.6)	
· Inadequate- n (%)	6 (4.1)	2 (2.4)	
Betalactamic more aminoglycoside - n (%) (%)aminoglycoside- n (%)	28 (19.6)	20 (24.1)	0.50
Betalactamic more quinolone - n (%)	79 (55.2)	44 (53.0)	0.78
Pa0_2_/FI0_2_ ratio - median (p 25–75)	177 (118–261)	180 (104–247)	0.41
Creatinine (mg/dl) - median (p 25–75)	1.20 (0.80–1.90)	1.50 (0.90–2.80)	0.03
Bilirubin (mg/dl) - median (p 25–75)	0.90 (0.46–1.55)	1.10 (0.50–2.50)	0.49
Leukocytes -median*10^3^/mm^3^ (p 25–75)	14.9 (10.0–20.4)	15.1 (8.7–20.4)	0.83
Lactic acid - median mmol/L (p 25–75)	2.00 (1.10–3.60)	3.50 (1.40–6.00)	<0.001
Platelets - median*10^3^/mm^3^ (p 25–75)	192 (131–273)	129 (77–219)	<0.001
INR - median (p 25–75)	1.27 (1.10–1.54)	1.41 (1.14–1.88)	0.01
aPTT - median seconds (p 25–75)	32 (28–41)	36 (29–46)	0.006
SOFA score - median (p 25–75)	9 (7–11)	11 (9–15)	<0.001
APACHE-II score - median (p 25–75)	19 (14–22)	23 (18–28)	<0.001
MDA - median nmol/mL(p 25–75)	2.89 (2.04–4.05)	3.93 (2.45–7.37)	0.002
TNF-alpha median pg/ml (percentile 25–75)	30 (20–50)	39 (18–75)	0.41
IL-10 - median pg/ml (percentile 25–75)	11 (5–37)	40 (8–138)	0.004

COPD = chronic obstructive pulmonary disease; PaO_2_/FIO_2_ = pressure of arterial oxygen/fraction inspired oxygen; aPTT = Activated partial thromboplastin time; INR = International normalized ratio; APACHE-II = Acute Physiology and Chronic Health Evaluation-II; SOFA = Sepsis-related Organ Failure Assessment; TNF = Tumor necrosis factor; IL = Interleukin; data are presented as number (percentage) or median (interquartile range).

Correlations of MDA serum levels with lactic levels, age, APACHE-II, SOFA, platelets, INR, aPTT, TNF-alpha and IL-10 are shown in Table 3. MDA serum levels positively correlated with lactic acid, SOFA, APACHE-II, INR, aPTT, TNF-alpha and IL-10, and negatively with platelet count.

**Table 3:** Correlation of MDA serum levels with lactic acid, SOFA, APACHE-II, age, coagulation markers and interleukins in severe septic patients.

	MDA serum levels
Lactatemia (mmol/L)	rho = 0.26; P<0.001
SOFA score (punctuation)	rho = 0.40; P<0.001
APACHE-II score (punctuation)	rho = 0.24; P<0.001
Age	rho = 0.10; P = 0.06
Platelets	rho = -0.33; P<0.001
INR	rho = 0.35; P<0.001
aPTT	rho = 0.21; P = 0.001
TNF-alpha	rho = 0.36; P<0.001
IL-10	rho = 0.34; P<0.001

SOFA = Sepsis-related Organ Failure Assessment score; APACHE-II = Acute Physiology and Chronic Health Evaluation-II; INR = International normalized ratio; aPTT = Activated partial thromboplastin time; TNF = Tumor necrosis factor; IL = Interleukin; rho = Spearmańs rank correlation coefficient.

Cox regression analysis showed that MDA serum levels were associated with survival at 30 days (Hazard ratio = 1.05; 95% confidence interval = 1.009–1.091; p = 0.016) after controlling for age, lactic acid levels, APACHE-II and aPTT (Table 4).

**Table 4:** Cox regression analysis to predict survival at 30 days.

	Hazard Ratio	95% Confidence Interval	p-value
MDA serum levels	1.05	1.009–1.091	0.016
Age	1.02	1.000–1.035	0.055
Lactic acid	1.08	1.003–1.167	0.041
APACHE-II	1.04	1.007–1.076	0.018
aPTT	1.01	1.003–1.022	0.012

APACHE-II = Acute Physiology and Chronic Health Evaluation-II; aPTT = Activated partial thromboplastin time.

Kaplan-Meier survival analysis showed that patients with MDA serum levels higher than 4.11 nmol/mL had a lower probability of survival at 30 days (log-rank = 18.1; Hazard Ratio = 2.4 (95% CI = 1.49–3.94); P<0.001) than patients with lower levels (Figure 1).

**Figure 1:** Survival curves at 30 days using MDA serum levels higher or lower than 4.11 nmol/mL.

We performed a ROC analysis to determine whether MDA serum levels could be used to predict outcomes in septic patients, and found that the area under curve of the MDA serum levels to predict 30-days survival was 0.62 (95% CI = 0.56–0.69; P = 0.002) (Figure 2).

**Figure 2:** Receiver operation characteristic analysis using MDA serum levels as predictor of mortality at 30 days in septic patients.

## Discussion

To our knowledge, this study includes the largest series providing data on the oxidative state in patients with severe sepsis. The most relevant findings were: a) higher serum levels of MDA in survivin and non-surviving severe septic patients than in healthy controls, b) there was a correlation between MDA serum levels and several indicators of severity in sepsis, c) the non-surviving septic patients had higher MDA serum levels than the survivors, and d) MDA serum levels could be used to predict outcomes in septic patients. Taken together, these results indicate that alteration of the oxidative state may be of great pathophysiological significance in septic patients.

We found that severe septic patients had higher serum levels of MDA than controls. These findings are consistent with the results of other small series with only 12 patients [3].

In our study, non-surviving septic patients had significantly higher MDA serum levels than survivors. These findings are consistent with the results of small series. Higher MDA serum levels have been reported in non-surviving than in surviving patients between 60 critically ill patients [13] and also specifically between 12 septic patients [3]; however, the sample size was too small to demonstrate that MDA serum levels are independently associated with survival in these series. The present study is the first to report that MDA serum levels could be used as a biomarker to predict the clinical outcome of septic patients. The large sample size, compared to previous studies, allowed us carried out a regression analysis to determine the independent contribution of MDA on the prediction of 30-day mortality. The imbalance favouring the oxidant state in non-surviving patients could lead to an increase of free radicals and these may contribute to cellular dysfunction, organ failure and finally death [14], [15].

Interestingly, we observed a significant correlation between MDA serum levels and several indicators of severity in sepsis, including lactic acid, APACHE-II and SOFA scores, and biomarkers of coagulation. Previous studies have reported a positive correlation between MDA and severity in critically patients [13] and in diabetic patients [16].

The strengths of our study are that it was a multicenter study (which increases the external applicability of results to other similar units) and the large sample size (that allowed us to increase the accuracy of the parameters analysed with respect to previous studies). Certain limitations should be recognized, such as the fact that no analysis of MDA serum levels during follow-up was performed. Measuring other compounds of oxidant and antioxidant states would be desirable in order to better evaluate this balance.

From a therapeutic perspective, the development of modulators of antioxidant/oxidant state could be used as a new class of drugs for the treatment of severe sepsis. In rats the administration of melatonin has been shown to reduce MDA levels and increase the levels of other antioxidant compounds such as glutathione reductase (GSH) and superoxide dismutase (SOD) [17]–[19]. In patients, the use of melatonin has reduced MDA serum levels in asphyxiated newborns [20] and septic newborns [21], and in adult burn patients it has reduced MDA serum levels and mortality [22].

### Conclusion

The novel findings of our study on severe septic patients, to our knowledge the largest series providing data on the oxidative state, are that elevated MDA serum levels probably represent an unbalanced oxidant state and are related with poor prognosis in patients with severe sepsis.
